# Abnormal Function of Circulating Follicular Helper T Cells Leads to Different Manifestations of B Cell Maturation and Differentiation in Patients with Osteosarcoma

**DOI:** 10.1155/2022/3724033

**Published:** 2022-04-19

**Authors:** Gang Zhao, Jianxiao Liang, Jingjing Cao, Shanyong Jiang, Jianshu Lu, Baoen Jiang

**Affiliations:** ^1^Department of Traumatic Orthopaedics, Dongying People's Hospital, Dongying, Shandong, China; ^2^Department of Radiology, Dongying People's Hospital, Dongying, Shandong, China

## Abstract

**Objective:**

The objective of this study is to investigate the effect of dysfunctional circulating follicular helper T cells (Tfh) on B cell maturation and differentiation in patients with osteosarcoma (OS).

**Method:**

Data from 30 OS patients who underwent diagnosis and treatment in our hospital, as well as those of 30 healthy subjects (HC), were collected at the same time. Flow cytometry was employed to identify proportions of CD4+CXCR5+Tfh cells and Tfh cell subtypes Tfh17, Tfh1, and Tfh2 in the patient's peripheral blood. CD40 L and IFN*γ* levels were detected after stimulating Tfh cells with an influenza antigen; the positive rates of CD27 and CD38 in B cells were detected before and after coculture with Tfh cells. qRT-PCR was carried out for Blimp-1 expression in B cells, and ELISA was employed to identify the levels of IgM, IgG, and IgA in B cells and IL-2, IL-10, and IL-4 in Tfh cells before and after coculture.

**Results:**

The percentage of CD4+CXCR5+Tfh cells in OS patients' peripheral blood increased significantly. The Tfh cell ratio increased along with the TNM stage, and the Tfh cell ratio in OS metastasis patients is greater than that in nonmetastatic patients. In addition, Tfh2 and Tfh17 cells increased drastically in OS patients, and no meaningful change was seen in Tfh1 cells. CD40 L levels of Tfh cells in OS patients were less than those of the HC group, and IFN*γ* was substantially increased. After coculturing the OS group's B cells with Tfh cells, the CD27+ and CD38+ cells of B cells were drastically greater, and Blimp-1 expression was also significantly increased. In addition, the levels of IL-21, IL-4, and IL-10 of Tfh cells in the OS group and the levels of IgA, IgG, and IgM in B cells were significantly reduced after coculture.

**Conclusion:**

Dysfunctional Tfh in OS patients can severely inhibit B cell development, maturation, and differentiation.

## 1. Introduction

Osteosarcoma (OS), a common bone-derived solid tumor, usually has a high incidence of occurrence in the population of 10–25 years old, ranking first among primary malignant bone tumors, with about 5/100 million new patients diagnosed every year [1–4]; the prognosis is also relatively poor, and the patient's 5-year survival rate with nonmetastatic osteosarcoma cured with surgery is below 20% [5]. With OS chemotherapy's widespread use in the 1970s and 1980s, the patient's 5-year survival rate with OS without metastasis raised significantly from 20% to about 70%. However, the 5-year survival rate of OS with metastasis patients is still less than 20% [6, 7]. This is still a problem that needs to be solved in clinical practice. Thus, boosting research on OS pathogenesis is essential for improving OS treatment levels.

Recent studies have shown that OS patients primarily have a suppressed immune system, have a low immune-competent cell function, and are in an immune system imbalance state, allowing tumor cells to grow and metastasize easily [8–10]. Circulating follicular helper T cells (Tfh) are CXCR5-positive CD4+ T cells [11], a new type of T cell subset discovered in recent years. Studies have confirmed that Tfh cells are essential in regulating host humoral immune homeostasis. Their main function is to assist B cell differentiation in forming plasma cells and memory B cells [12–14]. Current studies have confirmed that Tfh cells participate in the pathogenesis of various tumors [15–17]. Studies have shown that PD-1/PD-L1-mediated inhibition of the Tfh cell function leads to a decrease in interleukin 21 (IL-21) in patients with OS [18]. However, the position and clinical significance of Tfh cells in OS remain vague. To this end, this study collected data from OS patients and healthy subjects to uncover the CD4+CXCR5+Tfh ratio in patients' peripheral blood (PB) and its effect on B cell maturation marker levels, aiming to reveal the influence the circulating Tfh dysfunction has on B cell maturation and differentiation in OS patients.

## 2. Materials and Methods

### 2.1. Tissue Samples

Data from 30 osteosarcoma patients (OS) diagnosed and treated in our hospital, as well as those of 30 healthy subjects (HC), were collected. None of the study subjects had other tumor diseases or autoimmune diseases or received or underwent radiotherapy, chemotherapy, or surgery. There was no significant difference in gender and age between the OS group and HC group. All 30 OS patients were diagnosed by histopathology; clinical, pathological, and follow-up data were complete. OS patients were separated into group I, group II, group III, and group IV according to TNM staging and divided into nonmetastasis group and metastasis group based on whether metastasis occurred or not. The Ethics Committee of Dongying People's Hospital has given approval for this study and complies with the ethical standards set by the Chinese Medical Ethics Committee. Informed consent was acquired from all patients.

### 2.2. Isolation of PB Mononuclear Cells

Ten milliliters of peripheral venous blood was collected from each OS patient and thoroughly mixed with an equal volume of RPMI1640 at room temperature. Within 3 hours, peripheral blood mononuclear cells (PBMCs) were separated using lymphocyte separation solution (MP Biomedicals, USA) and density gradient centrifugation [19]. The isolated PBMCs need to be counted under a microscope and then resuspended in 10% fetal bovine serum to reach the final cell concentration of 1×107 mL-1 for subsequent use.

### 2.3. Tfh Cell Sorting

Each of the 107 PBMCs was resuspended with 40 *μ*l magnetic-activated cell sorting (MACS) buffer and added to a 10 *μ*l CD4+ T cell biotin-antibody cocktail before being incubated in the dark at 4°C for 5 min, rinsed with 1 ml MACS buffer, and centrifuged at 1,500 r/min for 5 min, and the supernatant was discarded. After resuspending the cells in 30 *μ*l MACS buffer, 20 *μ*l CD4+ T cell microbead cocktail was added, and the mixture was incubated in the dark at 4°C for 10 min before adding 1 ml MACS buffer to wash and centrifuge for 5 min at 1,500 r/min and dispose of the supernatant. Afterward, a sorting column (MS column), magnet block, and magnetic stand were placed; the column was wetted with 500 *μ*l MACS buffer, and 500 *μ*l MACS buffer was applied to resuspend the cells. After passing the cell suspension through the column, the effluent was gathered; 500 *μ*l MACS buffer was used to rinse the column 3 times, and the effluent was accumulated; the cell suspension was obtained 4 times and centrifuged at 1500 r/min for 5 min; the supernatant was removed, and the cells obtained are CD4+ T cells.

CD4 + CXCR5 + Tfh cells were labeled with FITC-CD4/APC-CXCR5 antibody [20]. FITC-CD4 and APC-55-CXCR5 dyes were included into the CD4+ T cells obtained above, and they were incubated for 30 min at 4 °C in the dark, rinsed with an accumulation of 1 ml FACS buffer, and centrifuged for 5 min at 1,500 r/min before discarding the supernatant; 200 *μ*l FACS buffer was used to resuspend the cells and transfer them to a sterile flow cytometer. The FACSAria flow cytometer (BD, USA) was turned on and adjusted to optimal working conditions for sorting the double positive CD4 and CXCR5. The collection solution was PBS containing 30% FCS; 106 cells were collected in about 20 minutes. A portion of the collection liquid was retained to test the purity of Tfh cell sorting, and the remaining portion was returned into the incubator for culture.

### 2.4. B Cell Isolation and Culture

B cells were labeled using CD19 antibody. A total of 107 PBMCs were resuspended with 90 *μ*l of MACS buffer; the solution was mixed well, 10 *μ*l of anti-CD19 microbeads was added, and the bottom of the tube was tapped for mixing. This was then incubated for 15 min at 4°C in the dark before washing the cells with the addition of 1 ml buffer and centrifuging it at 300 g for 10 min. The supernatant was discarded, and 1 ml buffer was added to resuspend the cells. CD19 + B cells were sorted and collected using a MidiMACS sorter.

### 2.5. Detection of Tfh Cell Subtypes and B Cell Markers [21]

PBMCs were stained with CD4-FITC, CXCR5-PE, CXCR3-APC, CCR6-PE, CD27-FITC, CD38-PE, CD40L-PE, and IFN*γ*-PE antibodies (BDPharmingenTM, USA) and incubated at 4°C for 30 min in the dark. After the antigen–antibody incubation was completed, the specimen was cleaned 3 times with 2.5 mL of flowing washing solution (Hyclone, USA)/PBS, then resuspended in 500 *μ*L of PBS, and put in storage at 4°C for performing upper flow cytometry analysis. The isotype control antibody was used to adjust the compensation of each channel and set the gate parameters. FlowJo software (Version 7.6.1, Tree Star Inc., USA) was employed to analyze the data obtained by flow cytometry. CD4+CXCR5+CXCR3+CCR6 indicates Th1-like cTfh cells, CD4+CXCR5+CXCR3-CCR6 indicates Th2-like cTfh cells, and CD4+CXCR5+CXCR3-CCR6+ indicates Th17-like cTfh cells.

### 2.6. Tfh Cell-Specific Antigen Reaction Detection

Influenza vaccine (0.1 *µ*g/mL) was added to PBMC (1 × 106 pcs/mL) along with an appropriate amount of GolgiStop and GolgiPlug (BD Company). The cells were cultured in a 37°C incubator for 6 hours. After removal, anti-CXCR5, anti-CD4, anti-CD3, and anti-CD40 L were employed for surface staining, and the cells were then permeabilized with Cytoperm/Cytofix; then anti-IFN*γ* was used to perform intracellular staining. After staining, the flow cytometer was used to perform fluid staining analysis to detect whether the patient's follicular helper T cells reacted to specific antigens and produced stimulating factors.

### 2.7. qRT-PCR

Cells were collected, and total cellular RNA was extracted with a total RNA extraction kit (Thermo Fisher Scientific, USA) and stored at −80°C. Then, cDNA was synthesized by reverse transcription following the cDNA reverse transcription PCR kit (Takala, Japan) protocol. The cDNA was taken for the reaction according to the instructions of the real-time PCR reagent (Takala, Japan). Data analysis was carried out using the 2^-ΔΔCt^ method [22].  Table 1 illustrates the primer sequences.

### 2.8. ELISA

Corresponding ELISA reagents were used to detect the levels of IgM, IgG, IgA, IL-2, IL-10, and IL-4 in the culture medium, and the detection steps were carried out strictly following the detection reagent (Lianke, China) protocol.

### 2.9. Statistical Analysis

The experimental data were statistically analyzed using SPSS22.0 software. Evaluation between the two groups was completed with the *T*-test, and one-way analysis of variance (ANOVA) was used for multiple group comparisons. The results were presented as mean ± standard deviation (Mean ± SD), and a considerable variation in the data was indicated as *P* < 0.05.

## 3. Results

### 3.1. Increased Proportion of Tfh Cells in Osteosarcoma Patients

The number of Tfh cells in osteosarcoma patients was first quantified by flow cytometry. The findings revealed that the CD4+CXCR5+Tfh cell proportion in PBMCs in the OS group was significantly higher than that in the HC group (Figure 1). In addition, its proportion increased along with the TNM stage (Figure 1B). In addition, it was also found that the fraction of CD4+CXCR5+Tfh cells in patients with metastasis of osteosarcoma was greater than in patients without metastasis (Figure 1(c)).

### 3.2. The Proportion of Tfh2 and Tfh17-Like Tfh Cells Increased Significantly in Osteosarcoma Patients

Tfh1, Tfh2, and Tfh17 are the three subgroups of Tfh cells, and their subtypes were further tested. It revealed that in contrast with the HC group, there was a significant increase in Tfh2 and Tfh17-like Tfh cells in the OS group, but no considerable variation was seen in Tfh1-like Tfh cells between the two groups (Figure 2).

### 3.3. Alterations in the Levels of CD40 L and IFN*γ* in Tfh Cells in Osteosarcoma Patients

After stimulating Tfh cells with influenza antigens, the immune ability of Tfh cells in OS patients and HC group patients was examined. The results showed that compared with the HC group, the level of CD40 L in Tfh cells in the OS group was significantly reduced while the level of IFN*γ* was significantly increased (Figure 3).

### 3.4. Dysregulation of Tfh Cells in Osteosarcoma Patients Affects B Cell Maturation and Differentiation

Furthermore, through the coculture of B cells and Tfh cells, the effect of Tfh cells on the differentiation and maturation of B cells in osteosarcoma was identified. Outcomes demonstrated that IL-21, IL-10, and IL-4 levels in Tfh cells in the OS group were significantly reduced and the immune factors IgA, IgG, and IgM in B cells were also reduced considerably after coculture (Figure 4(b)). Before cocultivation, no meaningful deviation in Blimp-1 expression and CD27 and CD38 positive rates between the OS group and HC group were present. However, after cocultivation, the B cell Blimp-1 expression level and the CD27 and CD38 positive rate in the OS group were significantly less than those in the HC group (Figures 4(c) and 4(d)). This shows that dysregulation of OS patients' Tfh cells affects B cell maturation.

## 4. Discussion

OS is the greatest general bone primary malignant tumor in children and adolescents [23]. Current treatment methods for OS still mainly refer to the treatment criteria from 1970, that is, the comprehensive treatment of surgery and chemotherapy [24]. The latest advances in bioinformatics and science and technology have developed potential targets for the treatment of osteosarcoma. However, the clinical results have not been significantly improved [25]. Therefore, there is an urgent need to enhance the research of the biological characteristics and pathogenesis of OS in order to find new and effective treatment methods.

There is evidence that OS is an immunogenic tumor [26]. Due to the prominence of the immune system in OS disease progression, understanding the OS immune system is crucial in treatment optimization and prognosis improvement in patients [27]. Tfh cells are major effector T cell divisions, which play an important role in inducing antibody production and B cell differentiation [12, 28]. The expression of CXCR5 is the characteristic marker originally used to identify Tfh cells [29, 30]. Studies have found that CD4+T cells expressing CXCR5 in human PB, namely, CD4+CXCR5+T cells, have the same phenotype and function as Tfh cells, namely, circulating Tfh cells [20, 31]. Current investigations have revealed that the percentage of CD4+CXCR5+Tfh to CD4+T cells in the PB of patients with myasthenia gravis is considerably greater than that of healthy controls and there is a positive correlation between the percentage and the stage of the disease [32, 33]. The results of this analysis revealed that the CD4+CXCR5+Tfh cell ratio in the PB of OS patients increased considerably and there was a positive correlation with TNM staging. In addition, it was also discovered that the CD4+CXCR5+Tfh cell ratio in the metastasis group also increased significantly. According to the different expressions of CCR6 and CXCR3 on the surface of cTfh cells, it can be divided into the following three subtypes: CD4+CXCR5 +CXCR3-CCR6+ (Th17-like), CD4+CXCR5+CXCR3-CCR6- (Th2-like), and CD4+CXCR5+CXCR3+CCR6- (Th1-like) [30], among which Tfh17 and Tfh2 cells can induce primitive B cells to produce antibodies, while Tfh1 cells cannot activate B cells [20]. Studies have reported that these three subtypes appear to be disproportional in particular autoimmune diseases, including rheumatoid arthritis and systemic lupus erythematosus [34, 35]. However, it is unclear whether these three subtypes experience disproportion in patients with OS. In this study, it was discovered that the Tfh17 and Tfh2 ratio in OS patients increased significantly but no considerable variation in the proportion of Tfh1 cells amongst the two groups was found, suggesting the involvement of Tfh and B cell maturation in OS patients. In addition, after stimulating CD4+CXCR5+Tfh cells with an influenza antigen, it was found that the level of CD40 L in the OS group was significantly reduced and the level of IFN*γ* was increased considerably. These results indicate that the cTfh dysfunction in OS patients can lead to an imbalance in the ratio of the cTfh pressure-type, reduce CD40 L levels, and increase IFN*γ* levels.

The transcriptional regulator Blimp-1 is an important regulatory factor that regulates the differentiation of primitive CD4+ T cells into Tfh cells. It mainly inhibits BCL-6 mRNA expression, etc., indirectly inhibiting the differentiation of initial T cells into Tfh cells [36, 37]. In this study, the OS group's Blimp-1 expression was substantially lower than the HC group's. Studies have shown that alterations in the local microenvironmental cytokine concentration can affect cell differentiation, among which IL-21, IL-10, and IL-4 are the most important influencing factors [15, 36, 38]. The expression of these cytokines allows Tfh cells to migrate to the germinal center and offer support for the class conversion, differentiation, and growth of B cells. Tfh cells regulate B cells' antibody production, differentiation, and proliferation by secreting IL-21, IL-10, and IL-4. References [39, 40] have reported that these cytokines can also act directly on B cells, promote plasma cells to differentiate from CD27 + memory B cells, induce class switching recombination, and stimulate naive B cells with poor response to secrete IgA, IgG, and IgM plasma cells [39]. This study found that the levels of immune factors IgM, IgG, and IgA and anti-inflammatory factors IL-21, IL-10, and IL-4 in the OS group were significantly reduced, indicating that the Tfh dysfunction in OS patients would also reduce inflammatory factor and anti-inflammatory factor levels. It was further found that after CD4+CXCR5+Tfh cells were cocultured with immature B cells, the rate of CD27 and CD38 positive cells in the OS group and HC group increased significantly. Even then, that of the OS group was notably less than that of the HC group. It indicates that the Tfh cell dysfunction in osteosarcoma can prevent B cell differentiation and maturation.

According to recent studies on the tumor microenvironment, tumor invasion and metastasis mechanism, antitumor immune system, and malignant tumor immune checkpoints, the prognosis of some malignant tumors has been significantly improved. Therefore, immunotherapy is an increasingly attractive treatment option for OS patients. The main reasons for the lack of development of OS therapy include the rarity, heterogeneity, and lack of discovery of tumor-specific antigens in this type of cancer. This study found that the proportion of Tfh in PBMCs of patients with OS was significantly higher than that of HC group. The results suggest that Tfh cells may be crucial in the pathogenesis of OS. In order to better explore the role of Tfh cells in the development of OS disease, the study further analyzed the changes in the proportion of Tfh cell subgroups at different stages of OS patients. The proportion of Tfh gradually increased with the increase in the tumor stage, which indicated that Tfh had a close relationship with the development of OS disease and tumor infiltration and had a close relationship with the progression of OS disease. Therefore, further research on Tfh in OS disease is of great significance to explore new immunotherapy modalities for OS. For successful OS immunotherapy, the conditions for immune surveillance must be elucidated, tumor-specific antigens of OS must be discovered, and multicenter collaborative studies must be conducted.

The above-mentioned results are helpful to our understanding of the pathogenesis of osteosarcoma, but due to the limited sample size, the results of this study still need to be supported by data from a large-sample multicenter trial, and the specific mechanism of Tfh in OS also needs further research.

## 5. Conclusion

In summary, the Tfh dysfunction in OS patients can significantly increase the ratio of CD4+CXCR5+Tfh cells in PB CD4+T cells, and it is positively associated with TNM staging. In addition, Tfh in the PB of OS can severely inhibit B cell differentiation and maturation, indicating the importance of the participation of B cells and Tfh cells in OS. These results can provide a new therapeutic direction for OS treatment.

## Figures and Tables

**Figure 1:** Changes circulating Tfh cell proportion in Osteosarcoma patients. (a), Flow cytometry detected Tfh cell amounts in PBMCs of OS and HC patients, ^*∗∗∗*^*P* < 0.001; (b), Flow cytometry detected the quantity of Tfh cells in patients with different stages of OS, ^*∗∗*^*P* < 0.01 vs. Group I; (c), Flow cytometry detected the ratio of Tfh cells in OS with and without metastasis, ^*∗∗∗*^*P* < 0.001.

**Figure 2:** Subtype changes of Tfh cells in patients with Osteosarcoma. (a), Flow cytometry detected Tfh2 cell amounts in PBMCs of OS and HC patients; (b), Flow cytometry detected Tfh2 cell amounts in PBMCs of OS and HC patients; (c), Flow cytometry detected Tfh17 cell amounts in PBMCs of OS and HC patients.^*∗∗∗*^*P* < 0.001.

**Figure 3:** The levels of CD40 L and IFN*γ* in Tfh cells of two groups of patients via flow cytometry. (a), the levels of CD40 L in Tfh cells between HC group and OS group, ^*∗∗∗*^*P* < 0.001; (b), the levels of IFN*γ* in Tfh cells between HC group and OS group, ^*∗∗∗*^*P* < 0.001.

**Figure 4:** The effect of Tfh cells on B cell maturation and differentiation in Osteosarcoma patients. (a), ELISA detected the levels of IL-21, IL-10, and IL-4 in Tfh cells; (b), ELISA detected the levels of factors IgA, IgG, and IgM in B cells after co-culture; (c), qRT-PCR detected Blimp-1 levels in B cells after co-cultivation; (d), The levels of CD27 and CD38 in B cells after co-culture were identified by flow cytometry, ^*∗∗∗*^*P* < 0.001 vs. HC group.

**Table 1:** qRT-PCR primer sequence.

Gene name	Primer sequence
Blimp-1	F 5′-AACGTGTGGGTACGACCTTG-3′
	R 5′-ATTTTCATGGTCCCCTTGGT-3′

GAPDH	F 5′-ACCACAGTCCATGCCATCAC-3′
	R 5′-TCCACCACCCTGTTGCTGTA-3′

## Data Availability

The data used to support the findings of this study are available from the corresponding author upon request.
